# Statistically significant association of the single nucleotide polymorphism (SNP) rs13181 (ERCC2) with predisposition to Squamous Cell Carcinomas of the Head and Neck (SCCHN) and Breast cancer in the north Indian population

**DOI:** 10.1186/1756-9966-28-104

**Published:** 2009-07-18

**Authors:** Amit Kumar Mitra, Neetu Singh, Vivek Kumar Garg, Rashmi Chaturvedi, Mandira Sharma, Srikanta Kumar Rath

**Affiliations:** 1 Genotoxicity Laboratory, Toxicology Division, Central Drug Research Institute, Lucknow, Uttar Pradesh, India; 2 Lucknow Cancer Institute, Jiamau, Lucknow, Uttar Pradesh, India

## Abstract

**Background:**

Non-synonymous single nucleotide polymorphisms (SNPs) within vital DNA repair genes may cause reduction of activity leaving the genome unrepaired resulting in genomic instability and cancer.

**Materials and methods:**

The present endeavour involved study on the association of the SNP rs13181 (Lys751Gln/A18911C) in the Nucleotide Excision Repair (NER) pathway gene ERCC2 (excision repair cross-complementing rodent repair deficiency, complementation group 2) with the risks of Squamous Cell Carcinomas of the Head and Neck (SCCHN) and Breast cancer using a case-control based association study among 685 (400 controls and 285 SCCHN-affected cases) and 395 (227 normal healthy female controls and 168 breast cancer cases) ethnically-matched samples, respectively from north India using Polymerase Chain Reaction followed by Restriction Fragment Length Polymorphism (PCR-RFLP) analysis.

**Results:**

Results showed significant association of rs13181 homozygous mutant (CC) [Odds Ratio (OR) 4.412, 95% Confidence Interval (CI) 2.413 to 8.068], heterozygous (AC) (OR 2.086, 95% CI 1.246 to 3.492) and combined mutant (AC + CC) (OR 2.672, 95% CI 1.647 to 4.334) genotypes with predisposition to Breast cancer. Statistically significant increase in SCCHN risk was also associated with the mutant genotypes of rs13181 (ERCC2), viz. homozygous mutant (CC) (OR 1.680, 95% CI 1.014 to 2.784), heterozygous (AC) (OR 1.531, 95% CI 1.092 to 2.149) and combined mutant (AC + CC) (OR 1.560, 95% CI 1.128 to 2.158) genotypes.

**Conclusion:**

The results of this case-control study indicate that the polymorphism rs13181 might be a risk factor for predisposition towards SCCHN and breast cancer among north Indian subpopulations.

## Background

Cancer is a genetic disease resulting from gradual accumulation of changes in the DNA that activate proto-oncogenes and inactivate tumour-suppressor genes leading to genetic instability which is further aggravated by DNA damage and errors made by the DNA maintenance and repair machinery [1]. Many cancers are heritable due to inheritance of specific variant allele/polymorphic variants [2-5]. Recent advancements in cancer research have provided increasing evidences that cancer acts through the interplay of high-risk variants in a set of low- and medium-penetrance genes rather than a few high penetrance genes [6,7]. The ability to metabolize carcinogens or pro-carcinogens, repair DNA damage and control cell signalling and the cell cycle are important examples of low- and medium-penetrance genes fundamental to homoeostasis which is why most cancers, including Squamous Cell Carcinomas of the Head and Neck (SCCHN) and Breast Cancer are based on these main factors [8,9]. SCCHN is the 5^th ^most common cancer worldwide [9] with high mortality ratios among all malignancies accounting for 12% of all cancers in men and 8% of all cancers among women [10]. SCCHN are the commonest forms of cancers of the head and neck that start in the cells forming the lining of the mouth, nose, throat and ear or the surface covering the tongue. The major head and neck sites include the oral cavity, the pharynx (nasopharynx, oropharynx and hypopharynx), the tongue (anterior 2/3^rd ^and posterior 1/3^rd ^or base of tongue), the larynx and the paranasal sinuses. Breast cancer is the primary subtype of cancer leading to death among women in developing countries. 13% out of the 58 million deaths worldwide in the year 2005 were caused due to cancer which included 502,000 deaths per year due to breast cancer. Well-established risk factors ascribed to breast cancer include early menarche, late menopause, age of first child's birth, nulliparity and family history (FH) [11].

DNA repair is considered to play a key role in cancer susceptibility whereby some individuals are at very high risk of cancer due to SNPs in crucial DNA repair genes [12-15]. Inactivation or defect in DNA repair genes may be associated with increased cancer risk [16]. Genetic polymorphisms in DNA repair genes are very common events [17-19], and some studies have shown a significant effect of some of these polymorphisms in DNA repair capacity [20-22]. Evidence of inherited abnormalities in DNA repair genes and genes controlling carcinogen metabolism has been found to underline increase in risk of cancers [23].

The gene ERCC2 (located in the chromosomal location 19q13.3; OMIM ID 126340; Gene ID 2068; Gene length 18984) encodes the ERCC2/Xeroderma pigmentosum Type D (XPD) protein, which is one of the seven genetic complementation groups that forms an essential component of the Nucleotide excision repair (NER) pathway, a major DNA repair pathway that removes photoproducts from UV radiation and bulky adducts from a huge number of chemicals, cross-links and oxidative damage through the action of 20 proteins and several multiprotein complexes [13,24]. XPD is a highly polymorphic gene and correlation of its polymorphisms and cancer risk have been extensively studied [20,25]. Among the genetic polymorphisms in ERCC2, the SNP causing amino acid change in codon 751 (Lys to Gln) (SNP ID rs13181) have been considered very important and there is evidence that subjects homozygous for the variant genotypes of XPD have suboptimal DNA repair capacity for benzo(a)pyrene adducts and UV DNA damage [26,27]. The polymorphism rs13181 has been found to be functionally significant since studies have showed that it is associated with alterations in DNA repair efficiency [16,25,26,28-33]. Therefore, rs13181 has been studied for its role in various cancers as potential susceptibility factors [23,27,31,34-48], although no such report is available on the north Indian subpopulation cluster for the risks of SCCHN or Breast cancer.

In the present study, genetic association of the nonsynonymous SNP rs13181 with the risks of Breast cancer and Squamous Cell Carcinomas of the Head and Neck (SCCHN) was analysed using Polymerase Chain Reaction followed by Restriction Fragment Length Polymorphism (PCR-RFLP) in a subpopulation cluster-matched (Indo-European linguistic subgroup + Caucasoid morphological subtype) case-control based study among north Indians.

## Materials and methods

### Case and control sample collection

Blood samples (2 ml each) were collected following written informed consent from 168 Breast cancer patients and 285 SCCHN patients, following histopathological and cytological confirmation, from different parts of north India undergoing treatment at Lucknow Cancer Institute (LCI) and Sanjay Gandhi Post Graduate Institute of Medical Sciences (SGPGIMS) between September, 2005 and June, 2008. 400 (173 males and 227 females) unrelated ethnically-matched (linguistic and morphological subpopulation clusters) cancer-free blood donors from the north Indian states of Uttar Pradesh and Uttarakhand were included in the current study as healthy normal controls for cancer association studies. All the subjects inducted in this study belonged specifically to the Caucasoid morphological subtype [49] and Indo-European linguistic group [50] of north India. A questionnaire was filled by each subject providing information on gender, addiction (smoking, tobacco chewing, pan masala), race, ethnicity, education, religion, marital status, first-degree family history, history of benign disease, menopausal status (for women), etc. Information on tumour subtype, ER-PR status (for breast cancer patients), grading and stage of disease were obtained from medical records of the patients. All Breast cancer patients were non-smokers. The study was approved by Institutional Medical Ethics Committee of Central Drug Research Institute (CDRI).

### DNA Isolation from cancer samples

DNA was isolated from blood samples of SCCHN and Breast cancer cases and controls using QIAamp DNA Blood Midikit (Qiagen Inc.) following manufacturer's protocol, quantitated using spectrophotometer (Genequant pro, Amersham Biosciences) and stored at -20°C.

### Primer Designing and synthesis

Reference sequence of the gene ERCC2 and information on coding regions (CDS) were retrieved from NCBI's (National Center for Biotechnology Information) sequence databases. The primers 5' CCCCCTCTCCCTTTCCTCTGTTC 3' (Forward Primer) and 5' GGACCTGAGCCCCCACTAACG 3' (Reverse Primer) were designed for the present study on the SNP rs13181 (ERCC2) using PrimerSelect module of Lasergene v6.0 software (DNAStar). The primer sequences were verified using NCBI BLAST  and UCSC In-silico PCR  to eradicate the possibility of amplification of any non-specific DNA sequences and synthesized commercially.

### PCR Standardization and Amplification

Gradient PCR reactions were performed for standardization of DNA amplification conditions and optimization of annealing temperature for the set (forward + reverse) of primers. Briefly, the primer set was used to amplify a standard DNA template at different annealing temperatures (with increment of approximately 2°C) and the temperature at which highest amount of PCR product was formed (as visualised from agarose gel) was considered the optimum annealing temperature for further PCR reactions.

All PCR reactions were performed in 200 μl transparent PCR tubes (Axygen Scientific Pvt. Ltd.) on a peltier-based thermal cycler (PTC100, MJ Research) using reagents from Fermentas Life Sciences in a total reaction volume of 50 μl containing nearly 100 ng genomic DNA, 1.5 U Taq polymerase in 1× PCR buffer, 1.5 mM MgCl_2_, 0.2 mM dNTPs, and 15 pmol of each primer. Thermal cycling conditions were as follows: initial denaturation step at 95°C for 10 min, 31 cycles of PCR consisting of denaturation at 94°C for 1 min, annealing at 63.0°C for 1 min and extension at 72°C for 1 min, followed by a final extension step at 72°C for 5 min. The reaction was held at 4°C. The PCR products were visualized by electrophoresis on 1.2% agarose gel and stored at 4°C. For gel electrophoresis, 5 μl of the amplified product was mixed with 1 μl of 6× gel loading buffer (analytical grade water containing 30% glycerol, 0.25% bromophenol blue, 0.25% xylene cynole) and resolved on 1.2% agarose gel in TAE buffer at 85 volts for 1 1/2 hrs. 100 bp DNA markers (New England Biolabs) were run with the amplified products as reference.

### RFLP analysis for cancer association study

The restriction enzyme PstI (Fermentas Life Sciences) was selected for PCR-RFLP studies using SeqBuilder module of Lasergene 6.0 (DNAStar) and WATCUT , an on-line tool for SNP-RFLP analysis. The 413 bp PCR product was subjected to restriction digestion using PstI following optimum reaction conditions as per manufacturer's protocols. The digestion products were visualized by electrophoresis on 3% agarose gel for RFLP analysis and the genotypes were inferred from the number of bands observed in the gel. The homozygous wild type (AA) genotype generated a single band of 413 bp upon restriction digestion, the homozygous mutant genotype (CC) produced two bands of 322 bp and 91 bp, while the heterozygous genotype (AC) was inferred by the presence of all the three bands (413 bp, 322 bp and 91 bp) upon visualisation on agarose gel following restriction digestion using the enzyme PstI.

### Statistical Analysis for determination of genetic association

Maximum likelihood estimates of descriptive statistics like allele and genotype frequencies were calculated using Microsoft Excel. Further statistical analysis of data was performed using the computer softwares Statistical Package for the Social Sciences (SPSS) version 16.0 and GraphPad Prism version 5.0. Hardy-Weinberg Equilibrium (HWE) was tested online using Hardy-Weinberg Equilibrium Calculator  among cases and controls separately, comparing the observed allele counts with that of the expected, by means of Goodness-of-fit Chi square test at d_f _(degrees of freedom) = 1. 3 × 2 Contingency Chi-square test was performed to verify overall association of the genotypes between cases and controls. Odds ratios (OR), relative risk (RR) and corresponding 95% confidence intervals (CI) were estimated to ascertain association of individual genotypes with SCCHN and Breast cancer risks. Logistic regression was performed to calculate adjusted ORs for subsequent analysis of potential risk factors like gender, smoking, Tobacco chewing and pan masala. All statistical tests were two-sided.

## Results

### Breast Cancer

Genotype results were successfully obtained among 215 female controls and 155 breast cancer cases. Chisquare_HWE _for genotype distributions were 0.2488 among controls. Genotype and allele frequencies for the loci rs13181 (ERCC2) among Breast cancer cases and normal healthy female controls have been provided in Tables 1 and 2, respectively. Allele frequencies of mutant allele [C] were 38.1% in control group and 57.1% in breast cancer group. The corresponding 3 × 2 contingency Chisquare value was 24.39 (P < 0.0001) for the genotypes of rs13181 (ERCC2) which suggested an overall significant association between breast cancer incidences and genotypes for the loci rs13181 (ERCC2). Subsequent analysis concerned assessment of risks associated with individual mutant genotypes, WM (heterozygous), MM (homozygous mutant) and WM + MM (combined mutant) with the risk of breast cancer based on Odds ratio (OR), 95% Confidence Intervals (CI) and corresponding P values.

**Table 1:** Details of genotype frequencies of the SNP rs13181 (ERCC2) among normal female and breast cancer subjects.

**rs13181 (ERCC2)**				
	**Genotype Frequencies**			

	**Normal Female**		**Breast Cancer**	

**WW (AA)**	84	0.391	30	0.194

**WM (AC)**	98	0.456	73	0.471

**MM (CC)**	33	0.153	52	0.335

**WM+MM (AC+CC)**	131	0.609	125	0.806

	215		155	

[WW-homozygous wild type; WM-heterozygous; MM-homozygous mutant]

**Table 2:** Details of allele frequencies of the SNP rs13181 (ERCC2) observed in normal female and breast cancer samples.

**rs13181 (ERCC2)**				
	**Allele Frequencies**			

	**Normal Female**		**Breast Cancer**	

**W (A)**	266	0.619	133	0.429

**M (C)**	164	0.381	177	0.571

	430		310	

[W-Wild type allele; M-Mutant allele]

Statistically significant association with breast cancer susceptibility was observed for the mutant genotypes of the polymorphism rs13181 in the gene ERCC2 viz. homozygous mutant (CC) (OR 4.412, 95% CI 2.413 to 8.068), heterozygous (AC) (OR 2.086, 95% CI 1.246 to 3.492) and combined mutant (AC + CC) (OR 2.672, 95% CI 1.647 to 4.334). Results of association studies between the mutant genotypes and breast cancer risk are represented in terms of corresponding Odds ratios in Table 3. The association with breast cancer did not vary greatly with menopausal status. Analyses stratified by tumour grading and ER-PR status did not seem to modify the risk of breast cancer among carriers (data not shown).

**Table 3:** Representation of genetic association of the SNP rs13181 in the gene ERCC2 with the risk of breast cancer in terms of odds ratios of mutant genotypes.

**Genotype**	**OR**	**95% CI (OR)**	**P Value**
			

**WM (AC)**	2.086	1.246 to 3.492	0.0056

**MM (CC)**	4.412	2.413 to 8.068	P < 0.0001

**WM + MM (AC+CC)**	2.672	1.647 to 4.334	P < 0.0001

[CI-Confidence Interval; OR-Odds Ratio; WW-homozygous wild type; WM-heterozygous; MM-homozygous mutant; WM + MM-combined mutant genotype

WW was considered as the referent category during the calculation of ORs.

An OR >1 denotes positive association, while OR <1 signifies protective/negative association with cancer risk.]

### Squamous Cell Carcinomas of the Head and Neck (SCCHN)

Genotype results were successfully obtained among 385 healthy unaffected control subjects and 275 SCCHN-affected cases for rs13181 (ERCC2). Chisquare_HWE _for genotype distributions was 0.345 among controls. The genotype and allele frequencies of the SNP rs13181 (ERCC2) among SCCHN cases and healthy control subjects are provided in Tables 4 and 5, respectively. Mutant allele frequencies were 34.4% among the controls and 41.1% among SCCHN cases. The corresponding 3 × 2 contingency Chisquare value was 7.417 (P = 0.0245) which implied an overall significant association between the prevalence of SCCHN and genotypes of the loci rs13181 (ERCC2). Subsequent analysis pertaining to the assessment of risks associated with individual mutant genotypes with regards to SCCHN risk depicted statistically significant association for rs13181 (ERCC2) homozygous mutant (CC) (OR 1.680, 95% CI 1.014 to 2.784), heterozygous (AC) (OR 1.531, 95% CI 1.092 to 2.149) and combined mutant (AC + CC) (OR 1.560, 95% CI 1.128 to 2.158) genotypes. Results of genetic association study with SCCHN risk presented in terms of crude odds ratios of mutant genotypes and adjusted odds ratios (AOR), adjusted for gender and habits like smoking, tobacco chewing and pan masala are shown in Table 6. Association of the selected SNPs with SCCHN risk did not vary greatly with tumour grading (data not shown).

**Table 4:** Details of genotype frequencies of the SNP rs13181 (ERCC2) among normal and SCCHN subjects.

**rs13181 (ERCC2)**	**Genotype Frequencies**			
	**Normal**		**SCCHN**	

**WW (AA)**	163	0.423	88	0.320

**WM (AC)**	179	0.465	148	0.538

**MM (CC)**	43	0.112	39	0.142

**WM+MM (AC+CC)**	222	0.577	187	0.680

	385		275	

[WW-homozygous wild type; WM-heterozygous; MM-homozygous mutant]

**Table 5:** Details of allele frequencies of the SNP rs13181 (ERCC2) observed in normal and SCCHN samples.

**rs13181 (ERCC2)**				
	**Allele Frequencies**			

	**Normal**		**SCCHN**	

**W (A)**	505	0.656	324	0.589

**M (C)**	265	0.344	226	0.411

	770		550	

[W-Wild type allele; M-Mutant allele]

**Table 6:** Representation of genetic association of the SNP rs13181 in the gene ERCC2 with the risk of SCCHN among north Indians determined in terms of odds ratios of mutant genotypes.

**Genotype**	**OR**	**95% CI (OR)**	**P Value**	**OR^a^**	**95% CI (OR^a^)**		**OR^b^**	**95% CI (OR^b^)**	
									

**WM (AC)**	1.531	1.092 to 2.149	0.0167	1.536	.816	2.892	1.297	.712	2.363

**MM (CC)**	1.680	1.014 to 2.784	0.0497	1.778	.692	4.567	1.446	.598	3.496

**WM + MM (AC+CC)**	1.560	1.128 to 2.158	0.0073	1.583	0.864	2.900	1.327	0.749	2.353

[CI-Confidence Interval; OR-Odds Ratio; WW-homozygous wild type; WM-heterozygous; MM-homozygous mutant; WM + MM-combined mutant genotype

WW was considered as the referent category during the calculation of ORs.

An OR >1 denotes positive association, while OR <1 signifies protective/negative association with cancer risk. OR^a^-Adjusted Odds Ratio for Gender, OR^b^-Adjusted Odds Ratio for Smoking, Tobacco chewing and Pan Masala]

## Discussion

The ERCC2/XPD protein functions as an ATP-dependent 5'-3' helicase joint to the basal TFIIH complex and participates in the local unwinding of DNA helix to allow RNA transcription machinery to access the promoter and to permit the NER machinery to access the lesion [51,52]. Several studies suggest that XPD protein may participate in the repair of ionizing radiation-induced oxidative damage [53,54]. The ERCC2 polymorphism, rs13181 located in exon 23, which consists of an A to C substitution in the coding region results in a Lys751Gln substitution in the important domain of interaction between XPD protein and its helicase activator, inside the TFIIH complex [55] which is indicative of a possible involvement of this SNP in defective activity of the gene.

Literatures evaluating the risk of rs13181 (ERCC2/XPD) polymorphism with the risk of Breast cancer have been controversial. Although some studies found no correlation between this polymorphism and breast cancer risk [39,56-59], significant association between rs13181 mutant (C) allele and overall breast cancer risk was found in some studies. While Terry et al observed a 20% increase in Breast cancer risk associated with genotypes having at least one variant allele (OR 1.21), both Terry et al and Bernard-Gallon et al observed a positive correlation of rs13181 heterozygous genotype with the risk of Breast cancer upon consideration of interactions between the mutant genotypes and anthropometric or lifestyle factors [60,61]. Correspondingly, the present study on the association of the SNP rs13181 with predisposition to Breast cancer showed a significant to highly significant positive association of greater than 2-folds for the rs13181 homozygous mutant (CC) (OR 4.412, 95% CI 2.413 to 8.068, P < 0.0001), heterozygous (AC) (OR 2.086, 95% CI 1.246 to 3.492, P = 0.0056) and combined mutant (AC + CC) (OR 2.672, 95% CI 1.647 to 4.334, P < 0.0001) genotypes.

On the other hand, only two studies have been found to have been conducted so far on the assessment of the risk of SCCHN associated with rs13181 (ERCC2) mutant genotypes. Both of these studies exhibited significant positive association with SCCHN risk among non-Hispanic white subjects and the south Indian population, respectively [44,62]. Correspondingly, in the current study, a statistically significant 1.5 or more-fold increase in SCCHN risk was associated with all the mutant genotypes of rs13181 (ERCC2), viz. homozygous mutant (CC) (OR 1.680, 95% CI 1.014 to 2.784, P = 0.0497), heterozygous (AC) (OR 1.531, 95% CI 1.092 to 2.149, P = 0.0167) and combined mutant (AC + CC) (OR 1.560, 95% CI 1.128 to 2.158, P = 0.0073) genotypes. Odds ratios adjusted against gender or habits (smoking, tobacco chewing and pan masala) using logistic regression also corroborated with the findings made using crude odds ratios only in terms of association of these potential risk factors with significant SCCHN risk demonstrating a potential role of these factors towards SCCHN susceptibility

## Conclusion

The results of the present investigation indicate that the polymorphism rs13181 might be a risk factor for predisposition towards SCCHN and Breast cancer among north Indian subpopulations. The data generated from this study may have wide-ranging applications for further epidemiological and public health related research on the Indian population.

The degree of susceptibility to cancers is hypothesised to be the final product of a mishmash of high-risk genetic polymorphic variants or SNPs in a subset of medium and low penetrance genes like DNA repair genes which, even in the absence of the highly penetrant variant cancer-associated alleles, may increase the degree of susceptibility towards cancers a few fold thus having a major impact on the population incidence of cancer [19]. Therefore, further initiatives towards the discovery of cancer susceptibility SNPs in other genes involved in the NER pathway and the unravelling of the functional aspects of interactions between SNP alleles shall be highly beneficial to interpret these potentially meaningful differences that may be cancer-causing and should therefore be vital for revealing the probable synergistic effect of gene-gene and gene-environment interactions in cancer susceptibility.

## Competing interests

The authors declare that they have no competing interests.

## Authors' contributions

AKM conceived of the study, participated in sample collection, carried out the molecular genetic studies, performed PCR-RFLP analysis, conducted the statistical analysis and drafted the manuscript. NS participated in sample collection. VKG offered clinical support and provided cancer samples. RC and MS carried out histopathology on the cancer samples. SKR supervised the study, participated in its conception, design and coordination and reviewed the manuscript. All authors read and approved the final manuscript.
